The article "Tiotropium Bromide Attenuates Mucus Hypersecretion in Patients with Stable Chronic Obstructive Pulmonary Disease" was published in 2021. Journal: Comput Math Methods Med.

# Tiotropium Bromide Attenuates Mucus Hypersecretion in Patients with Stable Chronic Obstructive Pulmonary Disease

**DOI:** 10.1155/2021/1341644

**Published:** 2021-10-05

**Authors:** Suyun Yu, Caili Zhang, Zhijun Yan, Qingqing Fang, Xiwen Gao

**Affiliations:** ^1^Department of Respiratory Medicine, Minhang Hospital Affiliated to Fudan University, Minhang District Central Hospital, Shanghai 201199, China; ^2^Minhang Qibao Community Health Service Center, Shanghai 201108, China; ^3^Department of Gastroenterology, Minhang Hospital Affiliated to Fudan University, Minhang District Central Hospital, Shanghai 201199, China

## Abstract

**Background:**

Patients with stable chronic obstructive pulmonary disease (COPD) have been observed to benefit from tiotropium bromide. However, there are few studies of tiotropium bromide on sputum and sputum viscosity. To evaluate the effect of tiotropium bromide on mucus hypersecretion, a randomized, double-blind controlled trial was performed.

**Methods:**

120 cases of patients with pulmonary function grade II were divided into two groups, which include the treatment group given tiotropium bromide powder inhalation (18 *μ*g, inhalation, QD) and the control group given formoterol fumarate powder inhalation (12 *μ*g, inhalation, BID) plus ambroxol hydrochloride tablets (60 mg, oral, TID). After 3 months of treatment, the pulmonary function and *α*_1_-acid glycoprotein (*α*_1_-AGP) in sputum were detected, and the changes of glycoprotein and Ca^2+^ content were evaluated by Miller classification.

**Results:**

Three patients (2 cases in the treatment group and 1 case in the control group) were dropped due to loss of follow-up, and 117 cases of patients were enrolled in this study. After 3 months of treatment, the sputum character score, *α*1-acid glycoprotein, Ca^2+^ content, and lung function of the two groups were significantly improved; group comparison analyses revealed that there was no significant difference in the content of *α*_1_-AGP, Ca^2+^ in sputum, and lung function between the two groups (*P* > 0.05), but the improvement of sputum properties was significant (*P* < 0.05), and the treatment group was better than the control group (*t* = −2.77; *P* = 0.007).

**Conclusions:**

Inhaled tiotropium bromide can effectively inhibit the mucus hypersecretion in stable COPD patients, improve the sputum properties and lung function of patients, and improve the quality of life of patients.

## 1. Introduction

Practically, chronic obstructive pulmonary disease (COPD) is characterized by persistent respiratory symptoms and airflow restriction [1]. In China, the incidence of COPD is 8.6%, and the number of sufferers has surpassed 100 million, putting a significant economic and social strain on the country [2]. It is estimated that more than 5.9 million people die of COPD and its related diseases every year by 2060 [3] due to the limited treatment options [4] and alter the long-term decrease in lung function conclusively [5]. The majority of COPD medications on the market now are bronchodilators [6, 7] that offer clinical relief by removing reversible airway restriction, which is a common but not universal characteristic of COPD [5]. Inhaled long-acting bronchodilators (ILBs) in combination with inhaled corticosteroids (ICS) are now recommended for the maintenance treatment of moderate-to-severe COPD [5], such as formoterol fumarate powder inhalation plus ambroxol hydrochloride tablets. Patients with COPD, on the other hand, are frequently unresponsive to corticosteroids, and patients using this class of anti-inflammatory medicines may be at an increased risk of pneumonia [8]. The orally active PDE4 inhibitor roflumilast was recently launched as an anti-inflammatory medication for the treatment of COPD; however, it is only approved for use in severe patients and is dose-limited due to side effects, notably in the gastrointestinal tract [9]. As a result, new therapeutic methods for COPD therapy, as well as a variety of innovative bronchodilators, are required [10], and anti-inflammatory drugs [11] and bifunctional agents [12] are under development for the treatment of this disease.

The article "Tiotropium Bromide Attenuates Mucus Hypersecretion in Patients with Stable Chronic Obstructive Pulmonary Disease" was published in 2021. Journal: Comput Math Methods Med.

One of the main features of COPD is airway mucus hypersecretion, which presents clinically as a persistent cough and expectoration. Excess mucus clogs the airways, causing airflow restriction and increasing the risk of bacterial infection. This leads to worsening airflow restriction, decreased airway mucociliary transport, respiratory infection, and acute COPD exacerbations (AECOPD) [13, 14]. Formoterol fumarate is a long-acting *β*2-adrenergic agonist used to prevent COPD-induced bronchospasm [15]. Published studies have shown that formoterol fumarate has a rapid bronchiectasis effect [16], which may enhance compliance, and continue bronchiectasis within 12 hours, with a cumulative effect when inhaled twice a day. Ambroxol hydrochloride tablets are mainly suitable for patients with thick sputum that is not easy to cough up [17]. Studies have shown that after treatment with ambroxol hydrochloride tablets, the number of inflammatory cells and plasma TNF-*α*, IL-8, and IL-6 levels in COPD rats were significantly reduced after treatment, and lung tissue inflammation was reduced [18].

Tiotropium is a long-acting second-generation muscarinic receptor antagonist that works by blocking acetylcholine binding to the M1, M2, and M3 muscarinic acetylcholine receptors (mAChRs) in the lungs. The quaternary ammonium compound binds reversibly to M1 mAChRs of the nerve ganglia of the lung, M2 mAChR postganglionic nerve fibers of the lung, and M3 mAChRs of the smooth muscles and mucous glands of the lung when the patient inhales the drug as an inhalation spray or inhalation powder. When tiotropium binds to the M1 and M3 mAChRs, it prevents the influx of intracellular calcium from generating a cellular response in the respiratory airways by blocking Gq alpha-protein activation of the phospholipase C pathway [19]. Bronchodilation, decreased mucous gland secretions, decreased ciliary beat frequency, suppression of fibroblast proliferation, and a poorly known anti-inflammatory action in the lungs are all effects of tiotropium's anticholinergic effect on the respiratory airway [20–23]. However, tiotropium was reported to improve the lung function of COPD patients. There are few studies of tiotropium bromide on sputum and sputum viscosity. In this study, tiotropium bromide inhalation was used to observe the stable COPD patients with phlegm and mucus, and formoterol fumarate powder inhalation combined with ambroxol hydrochloride tablets were used as control. Our findings showed that inhaled tiotropium bromide could effectively inhibit the mucus hypersecretion in stable COPD patients and improve the sputum properties and lung function of patients, so as to improve the quality of life of patients.

The article "Tiotropium Bromide Attenuates Mucus Hypersecretion in Patients with Stable Chronic Obstructive Pulmonary Disease" was published in 2021. Journal: Comput Math Methods Med.

## 2. Materials and Methods

### 2.1. Main Equipment and Drugs

The main equipment and drugs used were as follows: automatic biochemical analyzer (Olympus AU2700), centrifuge (Eppendorf, Centrifuge 5804R), spiral oscillator, electronic balance (Mettler-Toledo Instruments Co., Ltd., Switzerland), phosphate buffer (PBS), dithiothreitol (DTT), *α*_1_-acid glycoprotein (*α*_1_-AGP) reagent, and supporting calibration solution (No. 2672, Landau Company, UK). The lung function instrument used was the Quark PFT4 Ergo.

### 2.2. Study Population

The study was carried out with patients recruited at the Department of Respiratory Medicine, Minhang Hospital Affiliated to Fudan University, where they attended periodic control visits for COPD. Recruitment was carried out from January 2019 to July 2019.

The inclusion criteria were as follows: outpatients aged between 40 and 82 years old, FEV1/FVC was less than 70% and FEV1 was less than 80% and greater than or equal to 50% after clinical diagnosis of COPD and bronchodilator use, clinically stable period reached 6 weeks or more after the last aggravation, patients with excessive phlegm and sticky phlegm, and COPD was divided into GOLD B [5].

The article "Tiotropium Bromide Attenuates Mucus Hypersecretion in Patients with Stable Chronic Obstructive Pulmonary Disease" was published in 2021. Journal: Comput Math Methods Med.

The exclusion criteria were as follows: patients who were suffering from other pulmonary diseases, such as bronchial asthma, pneumonia, bronchiectasis, and lung cancer; patients who were suffering from severe heart, liver, and kidney dysfunction; patients who were suffering from severe neuropsychosis; patients who were suffering from severe prostatic hyperplasia combined with urinary retention, angle closure glaucoma, etc.; pregnant or lactating women; patients who were using oral or inhalational preparations that contain anticholinergic drugs; and patients who were unable or unwilling to continue.

The study design was authorized by the Ethics Committee of Minhang District Central Hospital with respect to the guidelines of the Declaration of Helsinki. Each participant gave written informed consent to participate in the study.

### 2.3. Study Design

Pulmonologists and geriatricians recruited and selected patients according to the abovementioned inclusion criteria. Finally, a total of 120 patients with stable COPD were included, all of whom matched the diagnostic criteria of the guideline for the diagnosis and management of the chronic obstructive pulmonary disease.

These patients were randomly divided into two groups, the treatment group and the control group, with 60 cases, respectively. The treatment group was given tiotropium bromide powder inhalation (18 *μ*g, inhalation, QD) (Zhengda Tianqing Pharmaceutical Group Co.). The control group was given formoterol fumarate powder inhalation (12 *μ*g, inhalation, BID) (Zhengda Tianqing Pharmaceutical Group Co.) combined with ambroxol hydrochloride tablets (60 mg, oral, TID) (Boehringer Ingelheim Shanghai Pharmaceutical Co.). The sputum specimens were collected and lung function was examined before and after treatment.

### 2.4. Collection and Treatment of Sputum Samples

Sputum samples were collected according to routine requirements. All subjects were treated with a disposable sputum collector before treatment and 3 months after treatment, and at least 2-3 ml of deep sputum was collected. Sputum samples were collected by the same person from 8:00 AM to 9:00 AM.

Two to 3 ml sputum was added with 0.1% dithiothreitol (DTT), 4 times the volume of the sputum; then, the mixture was shaken for 15 min with a spiral oscillator, and then the same volume of PBS was added. Finally, the mixture was shaken for 5 min and centrifuged for 10 min at 3000 rpm. The supernatant was placed at -70°C for determination.

### 2.5. Assessment Methodology

#### 2.5.1. Subjective Indicators

For the clinical macroscopic observation of sputum characteristics, the standard is shown in Table 1, referring to Miller's classification.

The article "Tiotropium Bromide Attenuates Mucus Hypersecretion in Patients with Stable Chronic Obstructive Pulmonary Disease" was published in 2021. Journal: Comput Math Methods Med.

#### 2.5.2. Objective Indicators

For objective indicators, sputum *α*_1_-AGP and Ca^2+^ (its content increased with the increase of sputum viscosity) and a lung function test (operated by the same person) were used. The *α*_1_-AGP kit of this test was purchased from Randox (UK). It was used to detect the content of *α*_1_-AGP in the samples by immunoturbidimetry on an automatic biochemical analyzer. For the lung function test, the lung function of the patients was checked on the first day and after 90 days, which include checking FEV1/FVC and FEV1% of the predicted value (FEV1%). The test should be repeated twice, the high value should be taken, and the difference between the two tests should be less than 5%.

### 2.6. Statistical Analyses

The data were analyzed using SPSS 21.0 statistical software (SPSS Inc.); mean ± standard deviation (SD) was used to express the age, sputum, and pulmonary function score before and after treatment; and *t*-test was used to compare within and between groups. Test level is *α* = 0.05.

## 3. Results

### 3.1. Tiotropium Bromide and Formoterol Fumarate Combined with Ambroxol Hydrochloride Demographics

Pulmonologists and geriatricians recruited and selected patients according to the inclusion criteria. In our study, 120 patients with stable COPD were included who satisfied the diagnostic criteria of the guideline for the diagnosis and treatment of chronic obstructive pulmonary disease. Due to the loss of follow-up, there were 2 cases in the treatment group and 1 case in the control group who were dropped. Finally, a total of 117 patients were included in the study. No adverse events occurred in all cases. There were 58 patients in the treatment group, including 35 males and 23 females, aged from 43 to 82 years, with an average of 67.13 ± 6.11 years. There were 59 cases in the control group, including 39 males and 20 females, aged from 45 to 80 years, with an average of 67.98 ± 5.82 years. The baseline data of the two groups were comparable, and there were no among-group differences in gender and age index (Table 2).

### 3.2. Tiotropium Bromide Improves the Sputum Properties of Patients with COPD

To explore the effect of tiotropium bromide on sputum indexes, the sputum score, *α*1-acid glycoprotein, and sputum Ca^2+^ of the two groups were detected. As shown in Table 3, there were no statistically significant differences between the two groups in the sputum score (*P* = 0.554), *α*_1_-AGP (*P* = 0.476), and sputum Ca^2+^ (*P* = 0.213). After treatment, no matter in the treatment group or control group, all of the sputum indexes were improved obviously. Furthermore, we also compared the pharmacodynamic effects of tiotropium bromide and formoterol fumarate combined with ambroxol hydrochloride. The results showed that there were nonsignificant improvements in *α*_1_-AGP (*P* = 0.518) and sputum Ca^2+^ (*P* = 0.644), but positive effect estimates for sputum score (*P* = 0.007). Our findings demonstrated that tiotropium bromide could improve the chronic sputum production in COPD and the phenotype of those with chronic sputum symptoms, suggesting the novel function of tiotropium bromide in improving sputum properties.

The article "Tiotropium Bromide Attenuates Mucus Hypersecretion in Patients with Stable Chronic Obstructive Pulmonary Disease" was published in 2021. Journal: Comput Math Methods Med.

### 3.3. Tiotropium Bromide Improves the Lung Function of Patients with COPD

Next, we investigated whether the introduction of tiotropium bromide in stable-phase COPD patients could improve lung function, physical performance, and quality of life. Before treatment, all the COPD patients suffered from bronchiarctia, and there was no significant difference in FEV1/FVC and FEV1/predicted value between the two groups. After treatment, the FEV1/FVC and FEV1/predicted values in the two groups were significantly increased (*P* < 0.05). Moreover, we also compared the pharmacodynamic effects of tiotropium bromide and formoterol fumarate combined with ambroxol hydrochloride on lung function. After therapy, we discovered that there was no significant difference between the two groups (Table 4), indicating that tiotropium bromide worked just as well as formoterol fumarate combined with ambroxol hydrochloride in improving the lung function of patients with COPD.

## 4. Discussion

COPD is a common and frequently occurring disease of the respiratory system [24]. The incidence and mortality are increasing year by year. The pathogenesis is still unclear. Chronic cough, sputum, and obstruction of the airway lead to the continuous decline in lung function. The quality of life is declining. It has brought a great economic burden to society and families. The global initiative for the prevention and treatment of COPD (GOLD) 2020 [25] points out that inhalation therapy is the first choice for stable COPD, and inhaled bronchodilators play a particularly important role in controlling the symptoms of COPD.

The most important pathophysiological changes of COPD are airway obstruction and airflow limitation. Studies have shown that airway mucus hypersecretion can aggravate small airway obstruction and reduce ciliary clearance function [26], which is an independent risk factor for the condition and prognosis of COPD. How to effectively inhibit the high expression of mucin is an important part of COPD research. The innervation of airway secretory cells includes three neural pathways: sympathetic (adrenergic), parasympathetic (cholinergic), and nonadrenergic and noncholinergic (NANC) innervation. Cholinergic nerve innervates mucus movement and respiratory secretions. Release of acetylcholine cholinergic nerve activated submucosal gland cells and stimulated mucus secretion. This is because these two illnesses are characterized by mucus hypersecretion, and muscarinic agonists promote mucus production. Tiotropium bromide is a new type of anticholinergic drug, and formoterol fumarate inhibits cholinergic and NANC-induced contractions [27]. In this study, we found that after 3 months of treatment, the sputum trait scores, *α*1-acid glycoprotein, Ca^2+^ content, and lung function of COPD patients in the two groups were improved. Recent animal studies have shown that rhinovirus (HRV) increases the production of mucin in the differentiation medium of primary human bronchial epithelial cells (ALI-PBEC), while fluticasone and tiotropium bromide can reduce the production of mucin induced by HRV. Another basic study [28] showed that tiotropium bromide reduced NE-stimulated MUC5AC, but had no effect on IL-13-stimulated MUC5AC. These results may be due to the increased production of acetylcholine by IL-13. In asthma research [29], a high dose tiotropium bromide was used to treat acute and recurrent allergic asthma in mice. It was concluded that tiotropium bromide could effectively inhibit airway and parenchymal inflammation and mucus hypersecretion. Similarly, some researchers [30] used tiotropium bromide (18 *μ*g/d) to treat patients with airway mucus hypersecretion of DPB who did not respond to macrolide drugs. Some of the results after using tiotropium bromide are as follows: the visual analogue scale (VAS) score was significantly improved; FEV1 was significantly improved after 3 months of tiotropium bromide treatment; and cough, sputum, and dyspnea symptoms of macrolide-resistant DPB patients were improved. Experimental results show that the sputum properties of COPD patients treated with tiotropium bromide were significantly improved. The effect may be due to the inhibition of airway secretion by tiotropium bromide through its anticholinergic effect on submucosal glands.

The article "Tiotropium Bromide Attenuates Mucus Hypersecretion in Patients with Stable Chronic Obstructive Pulmonary Disease" was published in 2021. Journal: Comput Math Methods Med.

The deficiency of this study is that the sample size is small, and the COPD patients in group A, group C, and group D have not been observed. The next step is to expand the clinical observation sample and observation cycle, and deepen the mechanism of the effect of tiotropium bromide, on sputum hypersecretion, so as to provide a theoretical basis for the treatment of COPD.

Previous studies on COPD have focused on the bronchiectasis of anticholinergic drugs [31]. However, there are few studies on its function in sputum. The results of this study showed that after 3 months of treatment with tiotropium bromide, the indexes of sputum viscosity by naked eye observation and objective reflection showed the improvement of sputum viscosity in COPD patients, and the improvement of lung function. Considering its role in improving the characteristics of sputum, it is involved in the improvement of lung function.

## Figures and Tables

**Table 1:** The standard of clinical macroscopic observation of sputum characteristics.

Symptoms/signs	Grading standard			
	0 points (-)	1 points (+)	2 points (++)	3 points (+++)
Characteristics of sputum	Pure and transparent, nonmucinous sputum	A little purulent transparent sputum	Purulent mucus (purulent<2/3)	Purulent mucus (purulent≥2/3)
Difficulty of expectoration	No phlegm	Sputum is easy to cough up	Sputum is difficult to cough up	On difficult cough
Sputum volume	The amount of expectoration was less than 10 ml	The expectoration volume is 10~50 ml day and night	The expectoration volume is 50~100 ml day and night	The amount of expectoration was more than 100 ml day and night
Cough	No cough	Mild cough, does not affect normal life and work	Between mild cough and severe cough	Severe cough, frequent cough day and night, affect work and sleep

**Table 2:** Comparison of baseline data between the two groups.

Group	Cases	Sex ratio (M/F)	Age (years)		
			Min	Max	Average $\left(\bar{X}\pm S\right)$
Treatment	58	35/23	43	82	67.13 ± 6.11
Control	59	39/20	45	80	67.98 ± 5.82
Test statistics		*X* ^2^ = 0.206			*t* = −0.765
*P* value		0.65			0.446

**Table 3:** Comparison of sputum indexes between the two groups before and after treatment.

Group	Cases	Sputum score		*α*1-Acid glycoprotein		Sputum Ca^2+^	
		Before	After	Before	After	Before	After
Treatment	58	7.12 ± 2.5	3.98 ± 1.39	901.89 ± 176.53	517.24 ± 103.25	4.65 ± 1.52	2.93 ± 0.55
Control	59	6.89 ± 2.37	4.71 ± 1.45	871.18 ± 175.97	536.03 ± 116.26	4.39 ± 1.46	2.99 ± 0.76
*t* value		0.594	-2.77	0.715	-0.65	1.257	-0.462
*P* value		0.554	**0.007**	0.476	0.518	0.213	0.644

**Table 4:** Comparison of pulmonary function between two groups of COPD.

Group		FEV1/FVC		FEV1/predicted value	
		Before	After	Before	After
Treatment	58	52.39 ± 6.65	59.29 ± 7.24	59.51 ± 5.85	66.89 ± 5.70
Control	59	51.44 ± 5.64	58.83 ± 5.07	58.67 ± 5.63	65.98 ± 6.24
*t* value		0.838	0.399	0.79	0.825
*P* value		0.399	0.691	0.431	0.411

## Data Availability

All data analyzed during this study are obtained from published articles or are available from the corresponding authors on reasonable request.
